This article has been retracted.

# Antisecretory, Gastroprotective, Antioxidant and Anti-*Helicobcter Pylori* Activity of Zerumbone from *Zingiber Zerumbet* (L.) Smith

**DOI:** 10.1371/journal.pone.0121060

**Published:** 2015-03-23

**Authors:** Heyam Mohamed Ali Sidahmed, Najihah Mohd Hashim, Mahmood Ameen Abdulla, Hapipah Mohd Ali, Syam Mohan, Siddig Ibrahim Abdelwahab, Manal Mohamed Elhassan Taha, Loke Mun Fai, Jamuna Vadivelu

**Affiliations:** 1 Department of Pharmacy, Faculty of Medicine, University of Malaya, Kuala Lumpur, Malaysia; 2 Department of Biomedical Science, Faculty of Medicine, University of Malaya, Kuala Lumpur, Malaysia; 3 Department of Chemistry, Faculty of Science, University of Malaya, Kuala, Lumpur, Malaysia; 4 Medical Research Centre, Jazan University, Jazan, Saudi Arabia; 5 Department of Medical Microbiology, Faculty of Medicine, University of Malaya, Kuala Lumpur, Malaysia; University of Sassari, ITALY

## Abstract

**Background:**

*Zingiber zerumbet* Smith is a perennial herb, broadly distributed in many tropical areas. In Malaysia, it’s locally known among the Malay people as “lempoyang” and its rhizomes, particularly, is widely used in traditional medicine for the treatment of peptic ulcer disease beyond other gastric disorders.

**Aim of the study:**

The aim of the current study is to evaluate the gastroprotective effect of zerumbone, the main bioactive compound of *Zingiber zerumbet* rhizome, against ethanol-induced gastric ulcer model in rats.

**Materials and Methods:**

Rats were pre-treated with zerumbone and subsequently exposed to acute gastric ulcer induced by absolute ethanol administration. Following treatment, gastric juice acidity, ulcer index, mucus content, histological analysis (HE and PAS), immunohistochemical localization for HSP-70, prostaglandin E2 synthesis (PGE_2_), non-protein sulfhydryl gastric content (NP-SH), reduced glutathione level (GSH), and malondialdehyde level (MDA) were evaluated in ethanol-induced ulcer *in vivo*. Ferric reducing antioxidant power assay (FRAP) and anti-*H*. *pylori* activity were investigated *in vitro*.

**Results:**

The results showed that the intragastric administration of zerumbone protected the gastric mucosa from the aggressive effect of ethanol-induced gastric ulcer, coincided with reduced submucosal edema and leukocyte infiltration. This observed gastroprotective effect of zerumbone was accompanied with a significant (*p <0*.*05*) effect of the compound to restore the lowered NP-SH and GSH levels, and to reduce the elevated MDA level into the gastric homogenate. Moreover, the compound induced HSP-70 up-regulation into the gastric tissue. Furthermore, zerumbone significantly (*p <0*.*05*) enhanced mucus production, showed intense PAS stain and maintained PG content near to the normal level. The compound exhibited antisecretory activity and an interesting minimum inhibitory concentration (MIC) against *H*. *pylori* strain.

**Conclusion:**

The results of the present study revealed that zerumbone promotes ulcer protection, which might be attributed to the maintenance of mucus integrity, antioxidant activity, and HSP-70 induction. Zerumbone also exhibited antibacterial action against *H*. *pylori*.

## Introduction

Gastric ulcer is the most common digestive system disease affecting a lot of people worldwide and has sparked medical and global economic interest. Many factors are involved in the development of gastric ulcer, such as stress, habit of smoking, nutritional deficiency, ingestion of non-steroidal anti-inflammatory drugs, hereditary predisposition and infection by *H*. *pylori* [1]. Although there are many drugs currently used in the clinical field to manage gastric ulcer disease, the majority of them exhibit several adverse reactions. Thus, there is need to find out more effective and less toxic antiulcer agents [2]. The high focus on the herbal medicines and the pharmacological activities of their bioactive compounds has resulted in the discovery of numerous natural drugs or herbal extracts [3]. In particular, a large number of medicinal plants demonstrated anti-ulcer properties [4], with quite less cost and a wide range of safety margin[5].

The Zingiberaceae plant family is most abundant in Southeast Asia, and it is widely used in traditional medicine [6]. *Zingiber zerumbet* Smith is one of the Zingiberaceae species, characterized by its significant economic outcome, since it used as a spice and as traditional medicine [7]. The plant is widespread in several tropical countries such as India, Bangladesh, Malaysia, Nepal, and Sri Lanka [8]. The rhizomes of *Zingiber zerumbet* have been intensively studied and found to exhibit a wide range of pharmacological activities such as antipyretic, analgesic properties, anti-inflammatory, chemo-preventive activities [9], antinociceptive, antiulcer, antioxidant, anticancer, antimicrobial, antihyperglycemic, antiallergic and antiplatelet activities [3]. In Malaysia, *Zingiber zerumbet* is locally called “lempoyang” and the rhizomes of the plant are widely used as traditional medicine for the treatment of peptic ulcers [8, 9], stomach ache, diarrhoea, asthma, rheumatism and as an anti-inflammatory [3].

Zerumbone, a monocyclic sesquiterpene compound (2,6,10-cy-cloundecatrien-1-one, 2,6,9,9-tetramethyl-,(E,E,E)-), was reported as the predominant bioactive compound from the rhizomes of *Zingiber zerumbet* [7, 10]. Earlier toxicity study on zerumbone determined its LD 50 value is 1.84 g/kg [11]. Although, zerumbone showed selective cytotoxic activity towards certain cancer cell lines, however, it has no or less effect on normal cell line [7]. Many studies have been performed to elucidate the biological activities of zerumbone, demonstrated many pharmacological activities such as antinociciptive, anti-inflammatory, antitumor, antiproliferative and antiplatelet aggregation [3]. However, there was no report or investigation on its effect on gastric ulcer. Thus, in our continuous search for a natural antiulcer compound from Malaysian herbal medicines, we isolated zerumbone from the rhizomes of *Zingiber zerumbet* for gastroprotective study.

Many experimental gastric ulcer models have been created to examine and identify the causes of gastric mucosal injuries, among them the ethanol ulcer model. Ethanol-induced gastric tissue damage in experimental animals is the most common ulcer model, since it penetrates easily and rapidly into the gastric mucosa, mediating various pathological events result in ulcer formation. [12]. Therefore, ethanol ulcer model is the ideal ulcer model and extensively have been utilized for the assessment of new antiulcer compounds [13].

Despite the traditional use of *Zingiber zerumbet* as antiulcer medicinal plant, and to the best of our knowledge, there was no such data among the extensive search on this valuable rhizome to show it is gastroprotective mechanisms. Thus, this study was conducted to provide a scientific base for the use of *Zingiber zerumbet* rhizomes and to illustrate the possible mechanism(s) that might be involved in the antiulcer action of its main bioactive constituent, zerumbone.

## Materials and Methods

### Plant material and isolation of zerumbone compound

Zerumbone (Fig. 1) was isolated from the rhizome of *Zingiber zerumbet* (Voucher No. ZZ-2009-127) deposited at the Herbarium of the Laboratory of Natural Products, IBS, University Putra Malaysia, UPM Serdang, Malaysia. Pure zerumbone crystals were prepared according to the method reported earlier [7]. The purity of zerumbone compound was identified using HPLC and LC–MS, respectively.

**Fig 1:** Chemical structure of zerumbone.

### Drugs and chemicals

Omeprazole, griess reagent, TPTZ and DTNB were purchased from Sigma-Aldrich Chemical Co. Kuala Lumpur, Malaysia. ketamine and xylazine were purchased from Pet Arcade Co, Kuala Lumpur, Malaysia. All other used chemicals and reagents were of analytical grade.

### Animals

Disease-free Sprague-Dawley male rats (225–250 ± 5g) and their standard commercial feed pellets were purchased from the Experimental Animal Unit, University of Malaya, Faculty of Medicine, Institutional Animal care And Use Committee (FOM IACUC), Kuala Lumpur, Malaysia. All animals were kept under constant environmental temperature of 22°C, with 12 hrs light/dark cycles and free access to feed and distilled water. Rats were caged in groups of 2–3 each and left for one week as acclimatization period.

### Ethic statement

This study was presented to the institutional ethical review board (FOM IACUC) for approval, and the approval was granted (2013-10-8/FAR/R/HMAS). All *in vivo* experimental procedures were performed in sterile condition in the Experimental Animal Unit of FOM IACUC following their guidelines. All animals received humane care, according to the criteria outlined in the “Guide for the Care and use of Laboratory Animals” prepared by the National Academy of Sciences and published by the National Institute of Health, USA.

### Antisecretory study

The effect of zerumbone on gastric acid output was determined following the recommended method [14]. Sprague Dawley rats were assigned equally into four groups (n = 6). After 24 hrs fasting, the animals anesthetized using ketamine 50 mg/kg and xylazine 5 mg/kg then their abdomen was open, the stomach was exposed and the pylorus was ligated. Immediately after pylorus ligature, animals were received the treatments intraduodenally (5mL/kg b.w) according to the following grouping:

- Group-1 control (5% Tween 80 v/v)
- Group-2 standard (omeprazole 30mg/kg)
- Group-3 zerumbone (5 mg/kg)
- Group-4 zerumbone (10 mg/kg)

Following treatment, the abdomen was then sutured. The surgery procedure was accomplished without any unintended deaths of animals. After four hours of continuous observation and monitoring, all animals sacrificed using the CO_2_ chamber, the abdomen was opened to place another ligature at the oesophageal end, then all the stomachs were removed immediately and the gastric content was collected into tubes and centrifuged at 2000 ×g for 5 min and the gastric secretion volume (mL) was determined. The pH value of the gastric juice was recorded using a digital pH meter. The total acidity of the gastric juice was determined by titrating with 0.01 N sodium hydroxide using phenolphthalein as indicator. One mL of the gastric juice was transferred into 100 mL conical flask, 2 or 3 drops of phenolphthalein solution were added and the titration was preceded until a definite pink color appeared. The total volume of alkali added was noted. The total acidity (expressed as mEq/l) was calculated using the following formula:

Acidity=(volume of NaOH×Normality of NaOH×100/0.1)×mEq/l/100gm

### Gastroprotective study

The gastroprotective effect of zerumbone was determined against ethanol ulcer model. Sprague Dawley rats were divided randomly into five groups (n = 6). Overnight fasted animals were treated orally (5mL/kg b.w) as follows:

- Group-1 normal control (5% Tween 80 v/v)
- Group-2 ulcer control (5% Tween 80 v/v)
- Group-3 standard (omeprazole 20mg/kg)
- Group-4 zerumbone (5 mg/kg)
- Group-5 zerumbone (10 mg/kg)

One hour later, all groups, except for group-1, were received absolute ethanol (5mL/kg) [15]. After one hour of continuous observation and monitoring, all animal anetheized using Ketamine 50 mg/kg and xylazine 5 mg/kg prior to collect the blood samples via cardiac puncture into tubes. The blood samples then centrifuged for 10 min at 11,940 x g to get pure serum which was stored at −80°C prior to use later for biochemical analysis [16]. After that, all the rats sacrificed using the CO_2_ chamber. The stomach was immediately removed, opened along the greater curvature, washed by iced cold phosphate buffer solution (PBS), photographed by an inverted microscope with digital camera (BX60 Olympus) and subjected for the determination of gastric ulcer area (mm^2^) using the image J software [17]. The gastroprotective assessment was displayed as an inhibition percentage (I %) calculated by the following formula described by [18].

Inhibition percentage(I%)=((UAcontrol−UAtreated)/UAcontrol)×100%.

Thereafter, each gastric tissue was cut into pieces and processed for further histological and mechanistic studies.

### Measurement of gastric mucus content and serum biochemical parameters

Each Stomach was opened along the greater curvature and washed with iced cold phosphate buffer solution (PBS). Using a glass slide, the surface of the gastric mucosa was gently scraped off and the collected mucus was weighted using a precise electronic balance [19]. The collected animal serum samples were analyzed at University Malaya Medical Centre using Hitachi Auto-analyzer to evaluate changes in serum biomarkers.

### Histological evaluation

For histological evaluation, a small fragment from each stomach was fixed in 10% buffered formalin solution, Followed by tissue dehydration with alcohol and xylene. After the dehydration, each sample was embedded in paraffin wax, sectioned on slides at 5 μm with a Leica rotation microtome. Group of slides were stained with hematoxylin and eosin (H&E) according to the recommended method [20].

### Lesion scoring system

Histopathological analysis was made under an inverted digital camera BX60 Olympus and the image J software was used to characterize the histopathological alteration in the damaged area [17]. The results were graded according to the literature scoring system [21]. The microscopic scoring was as follows: epithelial cell loss (score: 0–3), edema in the submucosa (score: 0–4), hemorrhagic damage (score: 0–4), and the presence of inflammatory cells (score: 0–3). The maximum total score was estimated up to 14. The evaluation performed by a pathologist who was unaware and blinded to the treatment.

### PAS staining

in oreder to assess the effect of the compound on mucosal glycoprotein’s production, group of the prepared tissue sections were stained with commercial periodic acid Schiff base (PAS) following the manufacture instruction (Sigma Aldrich, Malaysia, Periodic Acid-Schiff (PAS) Kit). The positive glycoprotein site will appear as magenta color. Image J software was used for the determination of the positively stained area (μm^2^) [17].

### Immunohistochemistry

Immunostaining was performed using DAKO ARK (Animal Research Kit), Peroxidase (DAKO, Carpinteria, CA, USA), to investigate the immunohistochemical localization of heat shock protein-70 (HSP70 Mouse monoclonal antibody, IgG_2b_, 200μg/mL-1:100). The protein was purchased from Santa Cruz Biotechnology, Inc., California, USA. The positive antigen site will appear as brown color. Image J software was used for the determination of the positively stained area (μm^2^) [17].

### Preparation of gastric tissue homogenate

Small fragments of each stomachs were weighted and homogenized (10% w/v) in 0.1 mol/l PBS containing mammalian protease inhibitor cocktail. The homogenates were then centrifuged at 10000 x g for 15 min at 4°C. The clear supernatant was aliquot and stored in −80 ^o^ C prior to quantify the biochemical parameters in the gastric tissue homogenate: GSH, MDA, NP-SH and PG.

### Glutathione (GSH) levels

GSH content into the gastric homogenate (GSH nmol/g tissue) was estimated using Ellman procedure [22]. Aliquot from the prepared tissue homogenate was allowed to react with 5,5-ditiobis-2-nitrobenzoic acid (DTNB) and the absorbance was read on a spectrophotometer at 412 nm.

### Thiobarbituric acid reactive substance assay

Thiobarbituric acid reactive substance (TBARS) assay was used to estimate gastric content of MDA, where MDA is a direct index of lipid peroxidation level [23]. In brief and according to the recommended method [24], the gastric homogenate was added to a 0.126 mL solution containing 26 mM thiobarbituric acid, 0.26 M HCL, 15% trichloroacetic acid and 0.02% butaylated hydroxyltoluene. The mixture was incubated in a water bath at 95°C for 1 h. After cooling, the mixture was centrifuged at 3000 g for 10 min. The absorbance was read in a spectrophotometer at 532 nm and the results were expressed in μmol/g tissue MDA. Tetramethoxy propane was used as standard.

### Estimation of nonprotein sulfhydryls

Gastric Mucosal nonprotein sulfhydryls (NP-SH) (μmol/g of tissue) was measured according to the recommended method of [25]. In brief, Aliquot of 5ml of the stomach homogenate was mixed with a solution containing 4 ml of distilled water and 1 ml of 50% Trichloroacetic acid. The mixture was vortex for 15 min and centrifuged at 3000× g. 2 ml of supernatant was mixed with 4 ml of 0.4 M Tris Buffer at pH 8.9; 0.1 ml of DTNB (5,5 dithio-bis-(2-nitrobenzoic acid)) was added and the mixture was shaken. The Absorbance was recorded within 5 min after DTNB addition at 412 nm against a reagent blank with no homogenate.

### Estimation of prostaglandin E 2

Sample from the oxyntic gland area was taken by biopsy (about 100 mg), immediately from each animal of the treated groups after they were sacrificed to determine the mucosal generation of PGE_2_ by competitive enzyme immunoassay using enzyme immunoassay kit for prostaglandin estimation (Cayman Chemicals). The gastric mucosa of different treated groups was excised and homogenized in an ice-cold Tris/HCl buffer containing 50 mM Tris/HCl (pH 7.4), 100 mM sodium chloride, 1 mM calcium chloride, 1 mg/mL D-glucose and 28 μM indomethacin according to the method of [26]. The protein concentration of the homogenate was measured by the method of [27]. Homogenate was centrifuged at 12,000×g for 30 min at 4°C for the determination of PGE_2_ concentration. The supernatant was transferred in separate vial and kept at − 70°C until assayed. The concentration of PGE_2_ present in the supernatant was measured in duplicates with PGE_2_ enzyme immunoassay kit. The assay was performed in a total volume of 150 μL with the following components being added in 50 μL volumes: standards or homogenate, enzymatic tracer and specific antiserum. After 1 h incubation at room temperature on shaker, the plates were washed and 200 μL of Ellman's reagents were dispensed into each well. After 1 h, the absorbance at 412 nm for each well was measured. Results were expressed as ng of PGE_2_ per mg of protein.

### Ferric-reducing antioxidant power (FRAP) assay

To describe the total antioxidant activity of zerumbone, the Ferric-reducing antioxidant power (FRAP) assay was accomplished following the procedure described by [28]. In Brief, FRAP reagent was prepared freshly from acetate buffer (pH 3.6), 10 mM TPTZ (2,4,6-Tri(2-pyridyl)-s-triazine) solution in 40 mM HCl and 20 mM iron (III) chloride solution in proportions of 10:1:1 (v/v), respectively. 50 μl of the compound were added to 1.5 ml of the FRAP reagent in the dark. 4 min later the absorbance was recorded at 593 nm. The standard curve was constructed linear (R2 = 0.9723) using iron (II) sulfate solution (100–1000 μM) and the results were expressed as μM Fe (II)/g dry weight of the compound.

### In vitro anti-*Helicobacter pylori* activity

Two *H*. *pylori* strains NCTC 11637 (American Type Culture Collection *ATCC* 43504) and J99 (*ATCC* 700824) were cultured with brain heart infusion broth (BHI; Oxoid) supplemented with 10% horse serum (Invitrogen) incubated at 37°C in a humidified CO_2_ incubator (Forma Steri-Cycle) for 3 days. Minimum inhibitory concentration (MIC) was determined by a modified microtiter broth dilution method on sterile 96-well Polypropylene microtitre plates with round-bottom wells (Eppendorf). Briefly, zerumbone was dissolved and diluted in 5% DMSO to give a 10x working stock solution. *H*. *pylori* was diluted to a final concentration of 2 x 10^6 CFU/mL in culture medium. Aliquots of 10μL of zerumbone were added to 90μL of *H*. *pylori* in a well of the microtitre plate. Concentration of the compound ranged from 31.25 to 250 μg/mL. The microtiter plate was incubated for 3 days in a CO_2_ incubator. The plate was examined visually and measured using a microplate reader (Varioskan Flash) at 600 nm to determine the lowest concentration showing complete growth inhibition, which was recorded as the MIC. Minimum bactericidal concentration (MBC) as the lowest concentration without growth on a chocolate agar plate supplemented with 7% lysed horse blood. Wells containing *H*. *pylori* with 10 μL of 5% DMSO and BHI medium containing 250 μg/mL zerumbone were used as control and blanks respectively. The results were recorded in accordance with the Clinical and Laboratory Standards Institute [29].

### Statistical analysis

The statistical differences between groups were determined according to SPSS version 16.0 using ordinary one-way ANOVA followed by Dunnetts multiple comparison tests. Analysis and graphs were prepared with GraphPad Prism version 5.02 for Windows, GraphPad Software, San Diego California USA, www.graphpad.com. All tests were performed at least in triplicates, and the values were represented as mean ± S.E.M (standard error of the mean). A value of *P <0*.*05* was considered significant denoted by (*).

## Results

### Effect of zerumbone on gastric acid secretion

Intraduodenal administration of zerumbone at doses of 5 and 10 mg/kg b.w and omeprazole at 30 mg/kg to the experimental rats, immediately after pylorus ligature, were significantly *(p <0*.*05)* reduced the acid output of the gastric content secreted during a period of 4 h. Table 1 shows the statistical significant differences between treatment groups on gastric acid secretion compared to the control.

**Table 1:** Effects of zerumbone administered intraduodenally, on the biochemical parameters of gastric juice obtained from pylorus-ligature model in rats.

Treatment	Volume	pH	Total acidity
Ulcer control (5% Tween 80 v/v)	6.23 ± 0.30	2.61 ± 0.22	203.30 ± 6.10
Omeprazole (30mg/kg)	1.86 ± 0.15*	4.61 ± 0.32*	70.00 ± 4.65*
zerumbone (5 mg/kg)	2.05 ± 0.17 *	3.93 ± 0.11*	98.67 ± 3.30*
zerumbone (10 mg/kg)	1.93 ± 0.08*	3.83± 0.20*	85.00 ± 2.41 *

Results are mean ± S.E.M. (n = 6). Statistical comparison was performed using ANOVA followed by Dunnet’s test.

* *P <0*.*05* when compared to the control group.

### Gross evaluation

The results showed that animal pre-treated with zerumbone or omeprazole were considerably reduced ulcer area formation compared to the ulcer control group. Omeprazole at 20mg/kg b.w and zerumbone at doses of 5 and 10 mg/kg b.w were significantly *(p <0*.*05)* inhibited ulcer formation by 76.77%, 75.59% and 88.75%, respectively as shown in Table 2. Gross observation showed that zerumbone pretreated groups (Fig. 2D and 2E) or omeprazole group (Fig. 2C) were considerably have less gastric lesions to the gastric mucosa compared to the ulcer control group; where ethanol-induced intense gastric mucosal damage in the form of an elongated band of hemorrhages (Fig. 2B).

**Fig 2:** Gross evaluation. Macroscopic appearance of the stomach of experimental rats submitted to ethanol-induced gastric ulcer in different groups showed that the normal control group exhibited an intact stomach without lesion (group A), ulcer control group showed extensive lesions to the gastric mucosa appears as elongated bands of hemorrhage (white arrow) (group B), reference control group pretreated with omeprazole at 20 mg/kg showed mild injuries to the gastric mucosa as opposed to group B (group C). Whereas, rats pretreated with zerumbone at 5 and 10 mg/kg, (group D and E, respectively) showed moderate to slight injuries to the gastric mucosa as opposed to group B (magnification: 1.8 x). (n = 6).

**Table 2:** Observed ulcer area, inhibition percentage, mucus content and serum analysis of zerumbone against ethanol-induced gastric ulcer in rats.

Pre-treatment (mg/kg)	Ulcer area (mm ^2^)	Inhibition (%)	Mucus weight (g)	ALT(IU/L)	AST(IU/L)
Ulcer control	178.48 ± 11.04	NA	0.89±0.2	55.4±2.71*	292±2.15
Normal control	0	100	0.99±0.3	35.67±1.67*	227±6.81 *
Omeprazole 20	41.44 ± 1.01*	76.77	1.91±0.2*	37±2.08 *	274.67±3.01 *
Zerumbone 5	43.55 ± 2.00*	75.59	1.56 ±0.4 *	48.4±1.47 *	278.04±2.02 *
Zerumbone 10	20.07 ± 1.09*	88.75	1.78±0.1 *	38.75±1.58 *	271.6±6.22 *

NA; not applicable; AST, Aspartate transaminase; ALT, Alanine Aminotranferase. Data are expressed as mean ± S.E.M. (n = 6),

*p < 0.05; significant vs. ulcer control. Statistical analysis was performed using one-way analysis of variance (ANOVA) followed by Dunnett’t test for multiple comparison.

### Gastric mucus content and biochemical analysis

The ulcer control group showed the lowest content of gastric mucus; while zerumbone-pretreated groups were significantly *(p <0*.*05)* increased the mucus production compared to the ulcer control group (Table 2). On the other hand, the serum analysis showed that the ulcer control group had increased levels of liver enzymes (AST and ALT). However, zerumbone pretreatment significantly *(p <0*.*05)* reduced the elevated such parameters (Table 2).

### Histological evaluation

Histological observation to the ulcer control group stained by H&E showed extensive gastric lesions, submucosal edema and leukocytes infiltration (Fig. 3B). However, zerumbone pretreated groups have relatively better protection as seen by decreasing ulcer area, reduction or complete absence of edema and leukocytes infiltration and flattening of mucosal fold was also observed (Fig. 3D and 3E, respectively). Further, the histological evaluation of H &E-stained gastric mucosa in rat pretreated with the studied doses of zerumbone against ethanol ulceration was interpreted as lesion score using image J software for each group in Table 3.

**Fig 3:** Histological evaluations. Results showed the histological appearance of the gastric mucosa of the experimental rats in the normal control group displayed normal arrangement of the gastric epithelium and gastric gland in the mucosal region (group A). Histological appearance of the ulcer control group showed extensive disruption to the surface epithelium and hemorrhagic necrosis, penetrating deeply into the gastric mucosa (white arrow), and extensive edema and leukocyte infiltration in the submucosa (black arrow) (group B). However, the rats pretreated with omeprazole at 20 mg/kg (group C) or that pretreated with zerumbone at 5 and 10 mg/kg (group D and E, respectively) showed the improved histological appearance compared to the user control (H & E stain: 20x). (n = 6).

**Table 3:** Lesion score of rat gastric tissue pretreated with zerumbone against ethanol-induced gastric damage.

Pre-treatment	Hemorrhagic damage (score 0–4)	Edema (score 0–4)	Epithelial cell loss (score 0–3)	Inflammatory cells (score 0–3)	Total (scores 14)
Normal control (vehicle)	0	0	0	0	0
Ethanol ulcer control	4 (4–4)	3 (2–4)	3 (2–3)	2 (0–3)	12 (4–14)
Omeprazole 20 mg/kg	0 (0–2) *	2 (2–1)	2 (0–2)	0 (0–1) *	4 (2–5) *
zerumbone 5 mg/kg	1 (1–2) *	2(2–4)	2 (0–2)	0 (0–1) *	5 (0–9) *
zerumbone 10 mg/kg	1 (0–2) *	1(1–2) *	1 (0–1) *	0 (0–0) *	3 (2–6) *

Data are expressed as mean ± S.E.M. (n = 6),

*p < 0.05; significant vs. ulcer control. Statistical analysis was performed using one-way analysis of variance (ANOVA) followed by Dunnett’t test for multiple comparison.

### Pas staining

PAS staining showed that, omeprazole pretreatment at 20 mg/kg and zerumbone pretreatment at 5 and 10 mg/kg were resulted in the expansion of a substantially continuous PAS-positive mucous gel layer that lining the entire gastric mucosal surface observed as magenta colour (Fig. 4C, 4D and 4E, respectively). However, stomachs of animals in the ulcer control group didn’t exhibit this magenta color of PAS stain, indicating the deleterious effect of ethanol on gastric mucus (Fig. 4B). The histological evaluation of PAS-stain was Further, interpreted as positively stained area (μm^2^) using image J software for each group in Table 4. Thess findings denote the potential effect of zerumbone to conserve the gastric mucus against the deleterious effect of ethanol.

**Fig 4:** PAS staining. Results showed that the histological appearance of the gastric mucosa of the normal control group displayed ordinary gastric mucus content as appeared by the faint PAS stain to the mucus cells (group A). In contrast, ulcer control group showed the absence of the PAS stain and the complete depletion of the mucous layer (group B). Omeprazole pretreatment at 20 mg/kg showed intense PAS stain noted as a bright purple color in the mucus cells lining the gastric pits, due to the carbohydrate-rich and viscous mucus they secrete (group C). Zerumbone pretreatment at 5 and 10 mg/kg (group D and E, respectively) have gradually increased in the mucosal secretion of the gastric glands. The black arrow indicates the glycoprotein appear as magenta color (PAS stain: 20x), (n = 6).

**Table 4:** PAS- stained area in rat gastric mucosa pretreated with zerumbone against ethanol-induced gastric damage.

Pre-treatment	Stained Area (μm^2^) / Field	% Area
Ulcer control	2.57 × 10^3^ ± 0.28	2.80
Normal control	7.84 × 10^3^ ± 0.31*	8.35
Omeprazole 20mg/kg	15.57 × 10^3^ ± 0.28*	16.58
Zerumbone 5mg/kg	9.80 × 10^3^ ± 0.23*	10.34
Zerumbone 10mg/kg	14.55 × 10^3^ ± 0.28*	14.45

Data are displayed as mean ± S.E.M. (n = 6),

*p < 0.*05*; significant vs. ulcer control. Statistical analysis was carried out using one-way analysis of variance (ANOVA) followed by Dunnett’t test for multiple comparison.

### Immunhistochemical

Immunohistochemical staining showed the overexpression of HSP-70 proteins in the gastric tissue of animals pretreated with the study doses of zerumbone appeared by the intense brown color of the positively stained antigen (Fig. 5C and 5D), while the ulcer control group didn’t activate HSP-70 at all (Fig. 5A). The immunoreactivity of HSP70 was interpreted as a positive stained area (μm^2^) using image J software for each group in Table 5. The results indicates that the HSP-70 expression in zerumbone-pretreated group might be contributed to its observed gastroprotection effect.

**Fig 5:** Immunohistochemical localization of Hsp-70 protein. The results showed the insignificant HSP70 expression in the gastric tissue of rat in the ulcer control group (group A). However, microscopic observation detected overexpression of HSP70 protein in the gastric tissue of rats pretreated with omeprazole at 20 mg/kg (group B) and zerumbone at 5 and 10 mg/kg (group C and D, respectively). The antigen site appears as a brown color (IHC stain: 20x), (n = 6).

**Table 5:** Effect of zerumbone on HSP70 immunreactivity in rat gastric mucosa induced to develop ulcer by ethanol.

Pre-treatment	Stained Area (μm^2^) / Field	% Area
Ulcer control	-	0
Omeprazole 20mg/kg	11.41 × 10^3^ ± 0.29*	10.36
Zerumbone 5mg/kg	16.45 × 10^3^ ± 0.28*	14.69
Zerumbone 10 mg/kg	31.39 × 10^3^ ± 0.59*	28.96

Data are expressed as mean ± S.E.M. (n = 6),

*p < 0.*05*; significant vs. ulcer control. Statistical analysis was performed using one-way analysis of variance (ANOVA) followed by Dunnett’t test for multiple comparison.

### Effect of zerumbone on PGE2 synthesis

In this study, as displayed in Fig. 6A, zerumbone at both study doses (5 and 10 mg/kg) was significantly (p < 0.05) still able to preserve a high PGE_2_ level despite administration of ethanol, when compared to the ulcer control group, where ethanol produced a sharp drop in PGE_2_ level. This outcome indicates the likely implication of PGE_2_ in the protective action of zerumbone against ethanol ulceration.

**Fig 6:** Gastric homogenate contents. The results showed the effect of zerumbone on gastric tissue homogenate contents of (A) prostaglandin E2 (PGE2), (B) non-protein sulfhydryl compound (NP-SH), (C) glutathione (GSH) and (D) malondialdehyde (MDA) levels. Compared to the ulcer control group, zerumbone pre-treatment significantly *(p <0*.*05)* increased the level of PGE2, NP-SH, and GSH. Meanwhile the level of MDA was decreased. (*) Indicate the significant differences between treatment groups at *(p <0*.*05)* compared to the ulcer control group. The results are expressed as mean ± SEM, (n = 6) by ordinary one-way ANOVA with Dunnett’s multiple comparison tests using Graph Pad Prism version 5.

### Effect of zerumbone on NP-SH compounds level

The level of the NP-SH was decreased subsequently to the intragastric administration of ethanol without treatment in the ulcer control group. In contrast, zerumbone pretreatment at 10 mg/kg significantly *(p <0*.*05)* elevated NP-SH level in the pretreated group compared to the ulcer control group. However, zerumbone at 5 mg/kg produced weaker effects on the increased in NP-SH level (Fig. 6B). The results indicate the probable involvement of NP-SH gastric content in the gastroprotection effect of zerumbone in this study.

### Effect of zerumbone on GSH level

The GSH level was significantly decreased subsequently to the intragastric administration of ethanol without treatment in the ulcer control group than all the pre-treated groups. However, zerumbone pretreatment significantly *(p <0*.*05)* restored the depleted GSH level compared to the ulcer group (Fig. 6C). The results point to the possible involvement of this endogenous antioxidant in the experimental gastroprotective effect of zerumbone.

### Effects of zerumbone on lipid peroxidation

MDA is used as an indicator of lipid peroxidation [23]. The ulcer control group showed the higher MDA level than the other pretreated groups. However, zerumbone pretreatment significantly *(p <0*.*05)* decreased gastric MDA level compared to the ulcer group (Fig. 6D). The results showed the efficacy of zerumbone to enhance cellular antioxidant system, evidenced by the reduced level of lipid peroxidation, which may implicate in its gastroprotection action.

### *In vitro* antioxidant evaluation of zerumbone

Given that Zerumbone demonstrated antioxidant activity evidenced by increased GSH level and inhibiting TBARS formation, FRAP assay was performed to evaluate the free radical scavenging activity of the tested compound. Zerumbone exhibited FRAP value of 58.3 ± 2.08 and the result was well compared with ascorbic acid showed 215.5 ± 3.11. Thus, it seems that the antioxidant activity of zerumbone is through the enhancement of the cellular antioxidant pathway.

### *In vitro* anti-*Helicobacter pylori* activity

In our continuous investigation for the possible mechanisms underlying the observed gastroprotective effect of zerumbone in this study, the microtiter dilution method was performed to examine the antibacterial action of zerumbone against *H*. *pylori*. Zerumbone represents respective MIC value of 250 μg/ml against two *H*. *pylori* strains; *H*. *pylori* NCTC11637 and *H*. *pylori* J99.

## Discussion

In this study, zerumbone from *Zingiber zerumbet* demonstrated gastroprotective efficacy against ethanol ulcer model in rats. The pretreatment by the intragastric administration of zerumbone at 5 and 10 mg/kg was efficiently protected the gastric mucosa from the damaging effect of ethanol in a dose dependent manner and the following discussion is to identify the possible mechanism(s) involved.

It's well know that peptic ulcer disease arises from the imbalance between the mucosal protective factors and the aggressive factors [30] and many gastroprotective agents were found to improve the cellular integrated work to increase mucosal resistance or to decrease the aggressive factors [31]. Nowadays, the therapeutic strategy for peptic ulcer treatment is focused on either the suppression of gastric acid secretion or the enhancement of gastro-protective factors [32]. Thus, we assessed the effect of zerumbone on *in vivo* gastric acid secretion against the pylorus ligature model in rats. The model of pylorus ligature is charackterized by producing a surge in the gastric acid secretion and stasis of acid. Therefore, the pylorus ligature model is an ideal and common method used to investigate the possible alterations in the gastric acid parameters. [33]. In the current search, the intradudenal administration of zerumbone was found to reduce the volume and total acidity of gastric juice induced by the pylorus ligature. These alterations might probably be due to the antisecretory activity of zerumbone.

Ethanol ulcer model is the widely used *in vivo* experiment to assess the gastroprotective activity of different agents from botanical resources [5]. It was found that ethanol-induced gastric injuries by direct and indirect toxic effect through different pathophysiological pathways [34]. Experimentally, the intragastric administration of ethanol was recognized to produce elongated bands of hemorrhagic, extended submucosal edema, mucosal crumbliness, inflammatory cells infiltration and epithelial cell loss [35]. In our study, zerumbone was administered orally into rats and this pretreatment protect the gastric mucosa from the deleterious effect of ethanol in a dose-dependent manner and the results were well confirmed by the light microscopy of the histopathological examination.

It was evidenced that reactive oxygen species (ROS)are implicated in the pathogenesis of ethanol-induced gastric mucosal injury [35]. ROS have an essential physiological role in the cellular homeostasis. ROS are unpaired molecules generated as a normal products during the mitochondrial respiration and from the peroxisomes to catalyze different redox reactions within the living organisms. In some cases, ROS production is increasing for a defensive purpose in response to certain external stimuli, harmful diet and human disease [36]. Normally these produced ROS are neutralized by endogenous antioxidant cellular system such as glutathione (GSH) and superoxide dismutase (SOD). However, oxidative stress status will occur when ROS production accumulated and exceeded over the cellular antioxidant system or when the defensive system is not functioning well to neutralize those oxidants [37]. Consequently, oxidative stress can cause lipid peroxidation, cellular death and tissue damage [38]. Oxidative stress was recognized as one of the major pathogenic causes, which concerned with the induction and the aggravation of gastric ulcer [39]. It was established that oxidative stress and diminished of endogenous antioxidant molecules are implicated in the direct and immediate deleterious effect of ethanol-induced gastric mucosal damage [40]. Non-protein sulphydryl compounds (NP-SH) are one of the most important protective factors against oxidative stress induced gastric ulcer by detracting the deliberated ROS in different experimental models such as in the ethanol gastric ulcer model [40]. Thus, high gastric content of NP-SH was found to protect gastric mucosa from the deleterious effect of ethanol [41]. Previous studies showed that ethanol administration is accompanied by a drop of endogenous sulfhydryl compounds, particularly and the most importantly glutathione (GSH) [42]. Subsequently, the low gastric GSH level increased the rate of lipid peroxidation, which mediate gastric tissue damage [40]. Malondialdehyde (MDA) is the main end product of lipid peroxidation. Thus, measurement of gastric MDA level can estimate indirectly the level of lipid peroxidation [43]. Thus, considering the role of NP-SH and GSH as an endogenous antioxidants providing a cellular protection against oxidative damage and the significance of MDA as a lipid peroxidation marker, we evaluated the effect of zerumbone on NP-SH, GSH and MDA level in gastric tissue homogenate. The results showed that zerumbone was significantly restored the depleted NP-SH and GSH level and decreased MDA level due to ethanol administration, as opposed to the ulcer control group. These findings suggest the possible efficacy of zerumbone to enhance cellular antioxidant system, which may consider one of its gastroprotective pathways.

It is well known the essential role of heat shock protein (HSPs) as gastroprotective factors against various stimuli [44]. HSPs are functioning as stressor proteins; HSP70s in particular are the chief stressor proteins expressed to confirm cellular protection as they refold or getting rid of the damaged proteins [45]. They up-regulated in response to various internal or external stimuli such as oxidative stress among others. Many pure natural compounds were reported to demonstrate cytoprotection effect against oxidative damage due to their activities as HSPs inducers [46]. Evidences showed that many nontoxic HSP-inducers are beneficial to provide cellular protection against gastric ulcer [47]. In our study, zerumbone pretreatment significantly induced HSP70 expression in the ulcerated gastric tissue of the experimental animals, indicating the possible participation of HSP70 in the observed gastroprotection effect of zerumbone.

For more investigation, we assessed the antioxidant activity of zerumbone compound by it is *in vitro* effect in FRAP assay. The FRAP assay was commonly used to evaluate the antioxidant activity of different medicinal agents [48, 49]. Practically, the antioxidant compound served as a reducing agent by donating a hydrogen atom. Thus, the reducing capacity of an agent is a remarkable indicator of its antioxidant power [50, 51]. In the current study, zerumbone showed insignificantly reducing activity. Thus it could be hypothesized that zerumbone might promote gastroprotection activity possibly through indirect and cellular antioxidant pathway.

It is well known the fundamental role of prostaglandins (PGs), particularly PGE 2 and PGI 2, in modulating the integrity of gastric mucosal layers and a variety of cytoprotective factors [52, 53]. PGs plays a significant part in resisting gastric mucosal injury as they control gastric acid secretion, enhances gastric mucus and bicarbonate production [54], increases mucosal blood flow and prohibits the diffusion of ulcerative agents into the gastric mucosa [55]. Earlier studies demonstrated the gastroprotective action of PG against ethanol-induced gastric damage [56]. So, as to investigate if this defensive factor is concern in the gastroprotection promoted by zerumbone, PGE 2 enzyme immune assay was performed. The results showed that zerumbone significantly preserved the gastric mucosal content of PGE 2, indicating the possible involvement of PGs in zerumbone- mediate gastroprotection against ethanol ulceration.

The stomach is always exposed to harmful endogenous and exogenous substances. Therefore, it possesses many defenses mechanisms to protect itself from damaging and extensive injury [57]. One of these gastroprotective mechanisms, and the most importantly, the gastric mucus layer, which is served as the first defensive line and physical barrier against the caustic effect of gastric acid secretion due to it is viscous, elastic, adherent and transparent characteristics [58]. In addition, gastric mucus has scavenging activity against ROS, thus provide antioxidant protection to the whole gastrointestinal tract [59]. It was reported earlier that ethanol ulcer model is associated with diminished of the mucus barrier and bicarbonate secretion [60]. Practically, periodic acid-schiff (PAS) staining is the widely used histochemical procedure to investigate the presence of glycoproteins. The periodic acid oxidizes the diol functional groups in the mucus, result in the formation of aldehydes, which in turn react with the schiff base reagent which precipitate a purple-magenta color [61]. In our work, we found that the administration of ethanol in rats diminished the gastric mucus layer. Nevertheless, pretreatment with zerumbone was significantly prevented a decrease in mucus production, as established by the observed intense magenta color, which signify the defensive effect of zerumbone on gastric mucus layer. These results demonstrated the essential role of mucus as a defensive factor in the observed gastroprotection promoted by zerumbone. Taken into account the stimulatory effect of NP-SH [62] and PGE 2 [54] on character and gastric mucus synthesis, we hypothesized that those factors may be implicated and elucidated the positive impact of zerumbone on maintaining gastric mucus production.

*H*. *pylori* is the most prevalent bacterial infection, affecting approximately 50% of the population around the world. *H*. *pylori* is widely considered as the major causative factors in the pathogenesis of peptic ulcer disease [63]. The bacterium is gram-negative pathogen, characterized by the flagellated and spiral-shaped, can colonize in the gastric mucus layer and adhere to the epithelium, where it obtained its supplements. The microscopic examination on the infected individuals showed that *H*. *pylori* generated gastric mucosal damage what is most distinguished by the infiltration of chronic inflammatory cells [64]. The current therapeutic regimen for *H*. *pylori* treatment consists of triple medicines; two antibiotics (amoxicillin and clarithromycin or metronidazole) plus a proton pump inhibitor or bismuth. Although this protocol verifies high efficacy in *H*. *pylori* eradication, it demonstrates some obstacles such as antimicrobial resistance and the less convenience usage to the patients [65]. For these reasons, there is increasing need to explore new antimicrobial agents with high efficacy to overcome the mentioned drawbacks of the current regimen. Many researches were conducted to discover potent antimicrobial agents against *H*. *pylori* infection from the medicinal plant origin [66]. Recently, there was a scientific agreement to define the potent antibacterial agent is that one which demonstrated MIC value of less than or equal to 250 [67, 68]. In this study, the antimicrobial effect of zerumbone compound was examined against *H*. *pylori* using microtiter dilution method, and the results showed a remarkable MIC value equal to 250. Thus, given the importance to discover a compound of both gastroprotective and anti- *H*. *pylori* activities, we could declare a novel activity of this known and valuable compound to be a promising agent in the treatment of peptic ulcer with or without *H*. *pylori* infection.

## Conclusion

To sum up, our study has demonstrated that zerumbone from *Zingiber zerumbet*, exert gastroprotection activity against ethanol- induced gastric ulcer model in rats. The gastroprotective mechanisms of zerumbone may possibly assign to its effect on the enhancement and raising the complementary action of gastric mucosal protective factors, such as the significant increased in the endogenous antioxidant GSH accompanied by the reduction of lipid peroxidation level. Moreover, zerumbone increased NP-SH and PGE 2 contents, those may involved in the resulted increased gastric mucus production. Zerumbone also up-regulated the expression of HSP70 to the gastric mucosal tissue. The study as well established the antisecretory activity of zerumbone compound in the pylorus ligature model, which may augment the observed gastroprotection action. Furthermore, zerumbone showed significant antimicrobial efficacy against *H*. *pylori*. Our work affords scientific evidences to the observed gatroprotective activity of zerumbone compound, making it a promising antiulcer compound. However, bearing in mind the presented gastroprotective mechanisms, and even though zerumbone was not tested against other ulcer model, yet, other mechanisms may be implicated and their parts, still need to be elucidated.
